# Advanced Glycation End Products Induce Peroxisome Proliferator-Activated Receptor γ Down-Regulation-Related Inflammatory Signals in Human Chondrocytes via Toll-Like Receptor-4 and Receptor for Advanced Glycation End Products

**DOI:** 10.1371/journal.pone.0066611

**Published:** 2013-06-12

**Authors:** Ying Ju Chen, Meei Ling Sheu, Keh Sung Tsai, Rong Sen Yang, Shing Hwa Liu

**Affiliations:** 1 Institute of Toxicology, College of Medicine, National Taiwan University, Taipei, Taiwan; 2 Institute of Biomedical Sciences, National Chung Hsing University and Department of Education and Research, Taichung Veterans General Hospital, Taichung, Taiwan; 3 Department of Laboratory Medicine, College of Medicine, National Taiwan University, Taipei, Taiwan; 4 Department of Orthopaedics, College of Medicine, National Taiwan University, Taipei, Taiwan; University Medical Center Freiburg, Germany

## Abstract

Accumulation of advanced glycation end products (AGEs) in joints is important in the development of cartilage destruction and damage in age-related osteoarthritis (OA). The aim of this study was to investigate the roles of peroxisome proliferator-activated receptor γ (PPARγ), toll-like receptor 4 (TLR4), and receptor for AGEs (RAGE) in AGEs-induced inflammatory signalings in human OA chondrocytes. Human articular chondrocytes were isolated and cultured. The productions of metalloproteinase-13 and interleukin-6 were quantified using the specific ELISA kits. The expressions of related signaling proteins were determined by Western blotting. Our results showed that AGEs enhanced the productions of interleukin-6 and metalloproteinase-13 and the expressions of cyclooxygenase-2 and high-mobility group protein B1 and resulted in the reduction of collagen II expression in human OA chondrocytes. AGEs could also activate nuclear factor (NF)-κB activation. Stimulation of human OA chondrocytes with AGEs significantly induced the up-regulation of TLR4 and RAGE expressions and the down-regulation of PPARγ expression in a time- and concentration-dependent manner. Neutralizing antibodies of TLR4 and RAGE effectively reversed the AGEs-induced inflammatory signalings and PPARγ down-regulation. PPARγ agonist pioglitazone could also reverse the AGEs-increased inflammatory signalings. Specific inhibitors for p38 mitogen-activated protein kinases, c-Jun N-terminal kinase and NF-κB suppressed AGEs-induced PPARγ down-regulation and reduction of collagen II expression. Taken together, these findings suggest that AGEs induce PPARγ down-regulation-mediated inflammatory signalings and reduction of collagen II expression in human OA chondrocytes via TLR4 and RAGE, which may play a crucial role in the development of osteoarthritis pathogenesis induced by AGEs accumulation.

## Introduction

Osteoarthritis (OA) is a progressive degenerative joint disease with signs and symptoms of inflammation, including joint pain, swelling, and stiffness leading to significant functional impairment and disability in older adults [1]. Cartilage damage in OA is caused by the disruption of a shift in the balance between catabolic and anabolic capacities of chondrocytes. Catabolic activities of OA chondrocytes are related to the elevated release of cartilage degrading enzymes, such as matrix metalloproteinases (MMPs), while anabolic activities result in the productions of type II collagen and aggrecan [2]. Several risk factors including obesity, increasing age, trauma, genetic predisposition, and endocrine factors are known to affect the progression of OA [3]. Aging has been considered to be a major risk factor for OA [4]. Advanced glycation end products (AGEs) produced irreversibly by the non-enzymatic glycation of proteins have been observed to accumulate with aging in various organs, especially in articular cartilage [5], [6]. Accumulation of AGEs in cartilage chondrocytes shows the decreased proteoglycan and collagen synthesis, which leads to stiffness and brittleness of the articular cartilage [7]. Furthermore, AGEs can also up-regulate the production of MMPs that mediate cartilage degradation leading to the joint destruction [8]. In chondrocytes of OA, AGEs has been shown to trigger the expressions of interleukin (IL)-6 and IL-8 through receptor for AGEs (RAGE) [9]. Activation of mitogen-activated protein kinase (MAPK)-regulated NF-κB signaling was involved in this AGEs/RAGE-induced expressions of IL-6 and IL-8 in chondrocytes [9]. On the other hands, toll-like receptor 4 (TLR4) has been shown to be up-regulated in the diabetic kidneys that the up-regulation of TLR4 is associated with the TLR4 ligands AGEs and high-mobility group protein B1 (HMGB1) in diabetic nephropathy [10]. HMGB1 has also been found to induce the amplification of inflammation and angiogenesis through TLRs and RAGE [11]. However, the role of TLR4 and RAGE in AGEs-induced inflammatory signalings in human chondrocytes remains to be clarified.

Peroxisome proliferator-activated receptors (PPARs) are ligand-activated transcription factors and members of the nuclear hormone receptor superfamily [12], [13]. PPARγ was originally identified to play an important role in adipocyte differentiation and lipid metabolism [14], [15]. It has been shown that PPARγ signaling is involved in the metabolic disorders [16] and cardiovascular diseases [17]. PPARγ is known to be expressed in many cell types including immune cells, endothelial cells, synoviocytes, and chondrocytes [18]–[20]. PPARγ expression has been found to be decreased in human OA cartilage and down-regulated in IL-1β-treated chondrocytes [21]. PPARγ agonist pioglitazone has also been demonstrated to be capable of decreasing the progression of guinea pig OA [22]. Activation of PPARγ lead to the inhibition of various inflammatory signalings, such as COX-2, IL-1β, IL-6 and TNFα, and MMP-1 expression in monocytes as well as synoviocytes [18], [19]. PPARγ activators have ability to prevent the inflammation-induced expressions of iNOS, COX-2, and MMP-13 in human chondrocytes [20], [23]. AGEs has recently been shown to down-regulate PPARγ expression in rabbit chondrocytes [24]. However, little is known about the relationship among AGEs, RAGE, TLR4, and PPARγ in the pathogenesis of OA. Here, we tried to investigate the roles of PPARγ, TLR4, and RAGE in AGEs-induced inflammatory signalings in human OA chondrocytes.

## Materials and Methods

### Ethics Statement

The samples of cartilage specimens were collected with written approvals from the institutional Ethics Committee at National Taiwan University Hospital, Taipei, Taiwan, and also from the patients.

### Reagents

Anti-mouse and anti-rabbit IgG-conjugated horseradish peroxidase, rabbit polyclonal antibodies specific for RAGE, TLR4, IκBα and Histone H1 were purchased from Santa Cruz Biotechnology (Santa Cruz, CA, USA). Mouse monoclonal antibodies specific for COX-2, collagen II, NF-κB p65, phospho-JNK, JNK, phospho-ERK, ERK, phospho-p38MAPK, p38MAPK, PPARγ, β-actin, α-tubulin were purchased from Santa Cruz Biotechnology (Santa Cruz, CA, USA). Rabbit polyclonal antibody specific for phospho-IKKα/β (Ser^180/181^) and phospho-p65 (Ser^536^) were purchased from Cell Signaling (Danvers, MA, USA). Mouse monoclonal antibody specific for RAGE was purchased from R&D Systems (Minneaplis, MN, USA). MMP-13 and IL-6 ELISAs and mouse monoclonal antibody specific for TLR4 were purchased from eBioscience. NF-κB (p65) Transcription Factor Assay Kit was purchased from Cayman Chemical Company (U.S.A). SB203580, SP600125, PD98059, bovine serum albumin (BSA), pioglitazone, pyrrolidine dithiocarbamate (PDTC) and all other chemicals were obtained from Sigma-Aldrich (St. Louis, MO, USA).

### Isolation and culture of chondrocytes from human articular cartilage

Human articular chondrocytes were isolated from healthy femoral head articular resected cartilage specimens and obtained from 10 patients aged 50–76 years (mean age, 63.7±2.51 years) who were generally healthy undergoing joint replacement surgery. Cartilage pieces were minced finely, and chondrocytes were isolated by sequential enzymatic digestion at 37°C with 0.2% collagenase (type II; Sigma-Aldrich) for four hours in Dulbecco's modified Eagle's medium (DMEM; Gibco, Grand Island, NY). Isolated chondrocytes were filtered through 100 µM nylon filters. The cells were grown in the plastic cell culture dishes in 95% air–5% CO_2_ with DMEM medium, which was supplemented with 20 mM HEPES and 10% heat-inactivated fetal bovine serum (FBS), 2 mM glutamine, penicillin (100 U/ml), and streptomycin (100 µg/ml) (pH adjusted to 7.4). Experiments were performed using cells from passages 3–7. In experiments, chondrocytes were plated in 6-well plates in complete DMEM medium and serum-starved for 12 hours overnight and then treated with 5–100 µg/ml AGEs for various time intervals in the presence or absence of pharmacological inhibitors for MAPKs or NF-κB or neutralizing antibodies for RAGE or TLR4. Chondrocytes cultured without AGEs or with BSA alone were served as controls.

### Preparation of AGEs

BSA (1 mg/ml) was incubated under sterile conditions with D-glucose (1 mg/ml) in 0.2 M phosphate buffer (pH 7.4) at 37°C for 8 weeks. After incubation, AGEs were dialyzed against PBS for 24 hours to remove unbound sugars and filter-sterilized using a 0.22 µM Millipore filter (Millipore, Billerica, MA, USA). AGEs were identified by Ultraflex III MALDI-TOF/TOF (Bruker) and the AGEs protein concentration was measured by BCA protein assay.

### Cell viability assay

Cell viability was determined by 3-(4,5-dimethylthiazol- 2-yl)-2,5-diphenyltetrazolium bromide (MTT; Sigma) assay. After treatment of cells with or without AGEs or with BSA alone for 24 hours, cells were washed with PBS. MTT (0.2 mg/ml) was then added to each well and the mixture was incubated for four hours at 37°C. Culture medium was then replaced with an equal volume of DMSO to dissolve blue formazan crystals. After the mixture was shaken at room temperature for 10 minutes, the absorbance was measured at 550 nm.

### Measurement of IL-6 and MMP-13 productions

Human OA chondrocytes (1×10^6^/ml) cultured in 6-well plates were stimulated with or without AGEs for 24 hours in the presence or absence of pioglitazone. IL-6 and MMP-13 productions in the culture media were quantified by using the commercially available IL-6 or MMP-13 specific ELISA kits (eBioscience) according to the manufacturer's instructions. The plates were read at 450 nm.

### Western blot analysis

The cellular lysates were prepared. Equal proteins (20–40 µg) were resolved on SDS-PAGE and transferred to immobilon polyvinyl difluoride (PVDF) membranes. The blots were blocked with 4% BSA for one hour at room temperature and then probed with the primary antibodies against COX-2, HMGB1, IκB kinase (IKK)α/β, phospho-IKKα/β, IκBα, phospho-IκBα, p65, phospho-p65, TLR4, phospho-ERK, phospho-p38MAPK, phospho-JNK, collagen II, NF-κB p65, (1∶1000, Santa Cruz) overnight at 4°C. After three washes, the blots were subsequently incubated with the secondary goat anti-rabbit or anti-mouse antibodies conjugated with horseradish peroxidase (1∶1000) for one hour at room temperature. The blots were visualized by enhanced chemiluminescence using Kodak X-OMAT LS film (Eastman Kodak, Rochester, NY).

### Preparation of nuclear extracts and NF-κB activation measurement

The binding activity of NF-κB to DNA was measured in nuclear extracts using NF-κB (p65) Transcription Factor Assay kit (Cayman Chemical Company). In brief, cells were lysed in a hypotonic buffer on ice for 15 minutes and centrifuged for 30 seconds to pellet nuclei. Then the pellet was re-suspended in nuclear extract buffer on ice for 15 min. The lysates were centrifuged at 14,000 × g for 10 minutes, and supernatants containing the nuclear proteins were collected. NF-κB activation was measured according to the manufacturer’s instruction using 10 µg of nuclear protein per well. Following color development, absorbance was read at 450 nm within 5 minutes.

### Statistics

The results are presented as mean±SEM. Each experiment was performed four times or more to ensure reproducibility. The significant difference from the respective controls for each experimental test condition was assessed by one-way analysis of variance (ANOVA) and two-tailed Student's t-test. The difference is significant if the *P*-value is less than 0.05. Software used:SigmaPlot 10.0 and GraphPad Prism 5.

## Results

### AGEs induce inflammatory responses in human OA chondrocytes

Human OA chondrocytes were treated with increasing doses of AGEs (5, 25, 50, and 100 µg/ml) for 24 hours and no significant cytotoxic effect was found as compared with normal control or BSA control (Figure 1A). AGEs effectively induced the productions of MMP-13 and IL-6 (Figures 1B and 1C) and resulted in the reduction of collagen II expression (Figure 1D) in a dose-dependent manner. Moreover, AGEs significantly up-regulated the expressions of COX-2 (Figures 2A and 2B) and HMGB1 (Figures 2C and 2D) in a dose- and time-dependent manner. On the other hand, AGEs (50 µg/ml) markedly induced the phosphorylations of IKKα/β, IκBα, and NF-κB p65 (Figure 3A, 3B and 3C) and the degradation of IκBα (Figure 3B) and the translocation of NF-κB p65 from cytosol to nucleus (Figure 4A and 4B) in a time-dependent manner. Also, AGEs could significantly activate NF-κB activity. (Figure 4D). Pretreatment with NF-κB inhibitor PDTC (20 µM) could effectively reverse the reduction of collagen II expression induced by AGEs (Figure 3D). These results indicate that AGEs are capable of inducing inflammatory signalings and reducing collagen II expression in human OA chondrocytes.

**Figure 1:** AGEs induce inflammatory signalings in human OA chondrocytes. Human OA chondrocytes (1×10^6^/ml) were incubated with AGEs (5–100 µg/ml) for 24 hours and cytotoxic effect was determined by MTT assay (A). Productions of MMP-13 (B) and IL-6 (C) were quantified by the ELISA kits. Protein expressions of collagen II (D) were determined by Western blotting. Densitometric analysis for collagen levels corrected to β-actin is shown. All data are presented as mean ± SEM for three independent experiments. *: P<0.05 versus control.

**Figure 2:** AGEs induce inflammatory signalings in human OA chondrocytes. Human OA chondrocytes (1×10^6^/ml) were incubated with AGEs (5–100 µg/ml) for 24 hours (A, C) or 0.5–24 hours (B, D). Protein expressions of COX-2 (A, B) and HMGB1 (C, D) were determined by Western blotting. Densitometric analysis for COX-2 and HMGB1 levels corrected to α-tubulin is shown. All data are presented as mean ± SEM for three independent experiments. *: P<0.05 versus control.

**Figure 3:** AGEs activate NF-κB signaling in human OA chondrocytes. Human OA chondrocytes (1×10^6^/ml) were incubated with AGEs (50 µg/ml) for indicated time intervals. The phosphorylations of IKKα/β (A), IκBα (B) and p65 (C) and the degradation of IκBα (B) were determined by Western blotting. In D, Chondrocytes were pretreated with PDTC (20 µM) for 1 hour followed by treatment with AGEs for 2 hours. Protein expression of collagen II was determined by Western blotting. Densitometric analysis for p-IKKα/β, p-IκBα, IκBα, p-p65, and collagen II levels corrected to α-tubulin is shown. All data are presented as mean ± SEM for three independent experiments. *: P<0.05 versus control. #: P<0.05 versus AGEs alone.

**Figure 4:** AGEs activate NF-κB activity in human OA chondrocytes, which can be reversed by pioglitazone. Human OA chondrocytes (1×10^6^/ml) were incubated with AGEs (50 µg/ml) for indicated time intervals. The expressions of nuclear p65 (A) and cytosol IκBα degradation (B) were determined by Western blotting. In C, chondrocytes were pretreated with PDTC (20 µM) for 1 hour followed by treatment with AGEs for 2 hours. Protein expression of PPARγ was determined by Western blotting. Densitometric analysis for nuclear p65, cytosolic IκBα, and PPARγ levels corrected to Histone H1, α-tubulin, and β-actin, respectively, is shown. In D, chondrocytes (1×10^6^/ml) were pretreated with pioglitazone (10 and 50 µg/ml) for 1 hour followed by stimulating with AGEs (50 µg/ml) for 24 hours. NF-κB activity was measured using NF-κB (p65) Transcription Assay kit and quantified with a spectrophotometric plate reader at wavelengths of 450 nm. All data are presented as mean ± SEM for three independent experiments. *: P<0.05 versus control. #: P<0.05 versus AGEs alone.

### Involvement of TLR4 and RAGE in AGEs-increased inflammatory responses in human OA chondrocytes

It has been reported that TLR4 and RAGE are presented in articular cartilage and are increased with aging and OA [25], [26]. We next investigated whether RAGE and TLR4 are involved in AGEs-induced increase of inflammatory responses in human OA chondrocytes. With AGEs (5–100 µg/ml) treatment, the expressions of TLR4 (Figures 5A and 5B) and RAGE (Figures 5C and 5D) were up-regulated in a dose- and time-dependent manner. Moreover, pretreatment with neutralizing antibodies for TLR4 and RAGE could effectively suppress the AGEs (50 µg/ml)-increased COX-2 (Figures 5E and 5F) and HMGB1 (Figures 5G and 5H) expressions. Quentification and statistical analysis were performed in Figure 6. These results indicate that TLR-4 and RAGE are involved in the AGEs-up-regulated COX-2 and HMGB1 expressions in human OA chondrocytes.

**Figure 5:** Involvement of TLR4 and RAGE in AGEs-induced COX-2 and HMGB1 protein expressions in human OA chondrocytes. In A-D, human OA chondrocytes (1×10^6^/ml) were treated with AGEs (5–100 µg/ml) for 24 hours (A, C) or 0.5–24 hours (B, D). Protein expressions of TLR4 (A, B) and RAGE (C, D) were measured by Western blotting. In E–H, human OA chondrocytes (1×10^6^/ml) were pretreated with neutralizing antibodies of TLR4 (20 µg/ml) and RAGE (10 µg/ml) for 1 hour followed by treatment with AGEs (50 µg/ml) for 24 hours. Protein expressions of COX-2 (E, F) and HMGB1 (G, H) were determined by Western blotting. Results shown are representative of at least three independent experiments.

**Figure 6:** Densitometric analysis for TLR4, RAGE, COX-2, and HMGB1 levels. Values are corrected to α-tubulin or β-actin levels. All data are presented as mean ± SEM for three independent experiments. *: P<0.05 versus control. #: P<0.05 versus AGEs alone.

### AGEs down-regulate PPARγ expression via TLR4 and RAGE in human OA chondrocytes

Previous evidence suggested that PPARγ plays a crucial role in the development of OA progression [27]. The decreased expression of PPARγ in OA cartilage might result in the increased inflammatory and catabolic responses [21]. We next tested whether AGEs affect the expression of PPARγ and the involvement of TLR4 and RAGE in human OA chondrocytes. AGEs (5–100 µg/ml) effectively decreased the expression of PPARγ in a dose- and time-dependent manner (Figures 7A and 7B). Chondrocytes pretreated with NF-κB inhibitor PDTC showed no effect on AGEs-induced down-regulation of PPARγ expression (Figure 4C). Moreover, pretreatment with neutralizing antibodies for TLR4 and RAGE could effectively suppress the AGEs (50 µg/ml)-decreased PPARγ expression (Figures 7D and 7E). These results indicate that TLR-4 and RAGE are involved in the AGEs- down-regulated PPARγ expression in human OA chondrocytes.

**Figure 7:** AGEs down-regulate PPARγ protein expression in human OA chondrocytes. Human OA chondrocytes (1×10^6^/ml) were treated with AGEs (5–100 µg/ml) for 24 hours (A) or 0.5–24 hours (B). In C and D, human OA chondrocytes were pretreated with neutralizing antibodies of RAGE (10 µg/ml; C) and TLR4 (20 µg/ml; D) for 1 hour and then stimulated with AGEs (50 µg/ml) for 24 hours. PPARγ protein expression was measured by Western blotting. Densitometric analysis for PPARγ level corrected to β-actin is shown. All data are presented as mean ± SEM for three independent experiments. *: P<0.05 versus control. #: P<0.05 versus AGEs alone.

### PPARγ agonist pioglitazone reverses the AGEs-increased inflammatory responses in human OA chondrocytes

We next evaluated the effect of PPARγ agonist pioglitazone on AGEs-increased inflammatory responses in human chondrocytes. As shown in Figure 8, pioglitazone (10 and 50 µM) significantly reversed the AGEs (50 µg/ml)-increased MMP-13 (Figure 8A) and IL-6 (Figure 8B) productions. Moreover, AGEs-induced COX-2 and HMGB1 expressions could also be inhibited by pioglitazone (Figure 8C and 8D). Pioglitazone also inhibited the AGEs-down-regulated collagen II expression (Figure 8E). On the other hand, the AGEs-increased NF-κB activity could be decreased by pioglitazone (Figure 4D). These results provide the further evidence that PPARγ down-regulation is involved in the AGEs-induced inflammatory signalings and collagen II reduction in human OA chondrocytes.

**Figure 8:** Effects of pioglitazone on inflammatory signalings in human OA chondrocytes. Human OA chondrocytes (1×10^6^/ml) were pretreated with pioglitazone (10 and 50 µg/ml) for 1 hour followed by stimulating with AGEs (50 µg/ml) for 24 hours. Productions of MMP-13 (A) and IL-6 (B) were quantified by specific ELISA kits. Protein expressions of COX-2, HMGB1, and collagen II were determined by Western blotting (C). Densitometric analysis for COX-2, HMGB1, and collagen II levels corrected to β-actin is shown. All data are presented as mean ± SEM for three independent experiments. *: P<0.05 versus control. #: P<0.05 versus AGEs alone.

### Involvement of MAPK signaling in AGEs-induced PPARγ down-regulation

MAPK signaling pathway has been shown to be involved in the AGEs-induced IL-6 and IL-8 expressions in chondrocytes [9]. We next investigated whether MAPK signaling is involved in the AGEs-mediated PPARγ down-regulation and collagen II reduction in human OA chondrocytes. AGEs (50 µg/ml) effectively increased the phosphorylations of JNK and p38MAPK in a time-dependent manner (Figures 9A and 9B). Pretreatment with SP600125 (a selective inhibitor of JNK) and SB203580 (a specific inhibitor of p38MAPK) effectively reversed AGEs-induced PPARγ down-regulation and collagen II reduction (Figure 9C). Moreover, AGEs (50 µg/ml) slightly increased the phosphorylation of ERK at 0.5 h after AGEs treatment (Figure 10A). However, PD98059 (an ERK inhibitor) could not affect the AGEs-induced PPARγ down-regulation (Figure 10B) and collagen II reduction (Figure 10C). These results indicate that MAPK signaling including JNK and p38MAPK is involved in the AGEs-mediated PPARγ down-regulation and collagen II reduction in human OA chondrocytes.

**Figure 9:** Involvement of MAPK signaling in AGEs-induced PPARγ down-regulation and reduction of collagen II expression. Human OA chondrocytes (1×10^6^/ml) were incubated with AGEs (50 µg/ml) for 0.5–24 hours (A, B) or 24 hours (C). The phosphorylations of JNK (A) and p38MAPK (B) were determined by Western blotting. In C, chondrocytes were pretreated with SP600125 (10 and 20 µM) or SB203580 (1 and 10 µM) for 1 hour followed by treatment with AGEs for 24 hours. Protein expressions of PPARγ and collagen II was determined by Western blotting. Densitometric analysis for p-JNK, p-p38MAPK, PPARγ, and collagen II levels corrected to JNK, p38MAPK, β-actin, and β-actin, respectively, is shown. All data are presented as mean ± SEM for three independent experiments. *: P<0.05 versus control. #: P<0.05 versus AGEs alone.

**Figure 10:** ERK signaling is not involved in the effects of AGEs on chondrocytes. Human OA chondrocytes (1 ×10^6^/ml) were incubated with AGEs (50 µg/ml) for 0.5–24 hours (A) or 24 hours (B,). The phosphorylation of ERK (A) were determined by Western blotting. In B and C, chondrocytes were pretreated with PD98059 (10 and 20 µM) for 1 hour followed by treatment with AGEs for 24 hours. Protein expressions of PPARγ and collagen II was determined by Western blotting. Densitometric analysis for p-ERK, PPARγ and collagen II levels corrected to ERK, β-actin, and β-actin, respectively, is shown. All data are presented as mean ± SEM for three independent experiments. *: P<0.05 versus control.

## Discussion

AGEs are a group of compounds that are formed mainly via the Maillard reaction, which happens when reducing sugar reacts with macromolecules such as amino acids in proteins, lipids or DNA in a non-enzymatic way. Several studies suggested that accumulation of AGEs may be a mechanism for the age-related development of OA [5]–[7]. In patients with focal degeneration of cartilage, the increased levels of AGEs have been found in their healthy cartilage [28]. Moreover, AGEs formation has also been shown to be accelerated in diabetic patients [29]. Diabetes has recently been suggested to be an independent risk factor for OA [30], [31]. Previous studies have shown that PPARγ signaling plays a potent anti-inflammatory role by negatively regulating the expressions of several pro-inflammatory genes [18], [19]. Several studies have also found that PPARγ agonists can reduce the expression and synthesis of cartilage degradation products *in vitro* and *in vivo*, and suggested that activation of PPARγ is capable of reducing the progression of OA [22], [20], [27], [32]. In the present study, we demonstrated for the first time that AGEs down-regulate the PPARγ expression and induce the productions of IL-6 and MMP-13, which result in the reduction of the expression of type II collagen (major cartilage matrix macromolecules) in human OA chondrocytes. PPARγ agonist pioglitazone significantly inhibited the productions of IL-6 and MMP-13 and reversed the reduction expression of collagen II. These results suggest that PPARγ signaling plays an important role in AGEs accumulating human OA chondrocytes.

The maintenance of structural and functional integrity of articular cartilage is known to depend on the balance between catabolic and anabolic of matrix components. The doublet effects of AGEs on synthesis and degradation of matrix constituents implicate that extracellular matrix turnover in articular cartilage is affected by accumulation of AGEs [33]. Of various types of collagens, type II collagen is related to build up the structural backbone of the extracellular matrix in human articular cartilage [34]. The degradation of collagen II by interstitial collagenases, MMPs, has been demonstrated to be a crucial step resulting in the destruction of the joints in OA patients [35]. MMP-13 (collagenase-3) is an important enzyme that preferentially cleaves collagen II in OA cartilage [35]. Moreover, IL-6 and HMGB-1 are two important mediators of inflammation. IL-6 is a multifunctional cytokine with a wide range of biological activities, including mediation of acute-phase responses and effects on bone metabolism [36]. Patients with OA exhibits elevated IL-6 levels [36]. HMGB-1 is a ubiquitous cytokine acting as a potent promoter of inflammation. HMGB-1 has been considered to be an important trigger of arthritis [37]. It has also been reported that HMGB-1 is involved in the pathogenesis of cartilage destruction in OA [38]. In the present study, the results showed that AGEs not only induce the productions of MMP-13 and IL-6 and the reduction of collagen II, but also increase the expressions of COX-2 and HMGB-1 in human OA chondrocytes in a dose- and time-dependent manner. In addition, PPARγ agonist pioglitazone could also effectively reverse these AGEs-induced effects in human chondrocytes, indicating that AGEs interfere with the extracellular matrix turnover in cartilage may through a down-regulation of PPARγ.

TLRs are known to evolutionarily recognize the conserved products unique to microbial metabolism involved in innate immune responses and the pathology of a number of inflammatory diseases [39]. Previous study has revealed that TLR4 is capable of regulating the early onset of joint inflammation and cartilage destruction in a murine model of immune complex-mediated arthritis [40]. On the other hand, RAGE is a member of the immunoglobulin superfamily and involved in homeostasis, development, and inflammation. RAGE interacts with diverse ligands, including AGEs, several members of the S100 protein family, and HMGB1, which has been shown to be present in articular cartilage [8], [41]. Increased expression of RAGE has been suggested to be related to various acute and chronic inflammatory diseases including OA [42]. A recent report has shown that both TLR and RAGE signaling systems are activated in preterm birth and suggested that the interactions between TLR-mediated acute inflammation and RAGE-mediated chronic inflammation may contribute to increase the preterm birth risk [43]. The study of Qin et al. has also suggested that the cross-talk between TLR4 and RAGE contributes an increase in inflammatory signalings in macrophages [44]. In the present study, we used neutralizing antibodies for TLR4 and RAGE to investigate the roles of TLR4 and RAGE in AGEs-induced inflammatory signalings in human OA chondrocytes. Our data showed that AGEs can up-regulate both TLR4 and RAGE expressions in a dose- and time- dependent manner. Both neutralizing antibodies for TLR4 and RAGE effectively suppressed the AGEs-increased COX-2 and HMGB-1 expressions and reversed the AGEs-induced PPARγ down-regulation. These findings indicate that both TLR4- and RAGE-mediated inflammatory signalings implicate in the AGEs accumulation-related OA pathogenesis.

TLR ligands have been found to be capable of leading the activations of MAPKs and NF-κB in chondrocytes [45]. Several studies have shown that MAPKs signals (p38, JNK, and ERK) are activated and involved in the increased inflammatory signalings and MMPs expressions in AGEs (100–400 µg/ml)-treated chondrocytes [9], [46], [47]. In these studies, the authors found that SB202190 (p38 inhibitor) could inhibit the AGEs-induced responses in chondrocytes; however, the effects of SP600125 (JNK inhibitor) and PD98059 (ERK inhibitor) are controversial [9], [46], [47]. In the present study, we have found that AGEs (50 µg/ml) markedly enhance the phosphorylations of JNK and p38MAPK, but induce a slight and transient increase in ERK phosphorylation, in human OA chondrocytes. Specific inhibitors of JNK and p38MAPK, but not ERK, effectively inhibited AGEs-induced down-regulation of PPARγ and the reduction of collagen II. These results suggest that JNK and p38MAPK are involved in the AGEs-mediated down-regulation of PPARγ in human OA chondrocytes. This finding is consistent with the findings in IL-1β-treated human chondrocytes [21] as well as AGEs-treated rabbit chondrocytes [24]. Besides, we have also found that PDTC, a NF-κB inhibitor, is capable of inhibiting the AGEs-induced reduction of collagen II expression, but can not abolish the AGEs-induced PPARγ down-regulation in human OA chondrocytes. Moreover, pioglitazone could decrease the AGEs-increased NF-κB activity and collagen II reduction. These findings suggest that the destruction of collagen II by AGEs in human OA chondrocytes may be through a JNK/p38MAPK-activated PPARγ down-regulation-triggered NF-κB activation signaling pathway.

In conclusion, as indicated in Figure 11, our results demonstrated for the first time that AGEs induce the inflammatory signalings, productions of MMP-13 and IL-6, and collagen II reduction in human OA chondrocytes via a TLR4 and RAGE-regulated p38MAPK/JNK-activated PPARγ down-regulation-triggered NF-κB activation signaling pathway. In addition, these findings implicate that the accumulation of AGEs is correlated to the erosion of human OA cartilage and stimulates chondrocytes to produce more catabolic factors (MMPs and cytokines) and less anabolic factors (collagen II). The TLR4 and RAGE-regulated down-regulation of PPARγ is important in the net catabolic effect of AGEs on cartilage and may play a crucial role in the development of OA pathogenesis induced by AGEs accumulation. The clinical significance of these findings needs to be clarified in the future.

**Figure 11:** The proposed schematic representation of AGEs-induced inflammatory signalings and resulted reduction of collagen II expression mediated by the down-regulation of PPARγ via TLR4 and RAGE in human OA chondrocytes is shown.
